RETRACTED

# Monodispersed Copper(I)‐Based Nano Metal–Organic Framework as a Biodegradable Drug Carrier with Enhanced Photodynamic Therapy Efficacy

**DOI:** 10.1002/advs.201900848

**Published:** 2019-05-22

**Authors:** Xuechao Cai, Zhongxi Xie, Binbin Ding, Shuai Shao, Shuang Liang, Maolin Pang, Jun Lin

**Affiliations:** ^1^ State Key Laboratory of Rare Earth Resource Utilization Changchun Institute of Applied Chemistry Chinese Academy of Sciences Changchun 130022 P. R. China; ^2^ University of Chinese Academy of Sciences Beijing 100049 P. R. China; ^3^ University of Science and Technology of China No. 96, JinZhai Road, Baohe District Hefei Anhui 230026 P. R. China

**Keywords:** biodegradable, glutathione reduction, hypoxia therapy, metal–organic frameworks, type I photodynamic therapy

## Abstract

Photodynamic therapy (PDT) has emerged as an alternative treatment of cancers. However, the therapeutic efficiency of PDT is severely limited by the microenvironment of insufficient oxygen (O_2_) supply and overexpression of glutathione (GSH) in the tumor. Herein, a biodegradable O_2_‐loaded CuTz‐1@F127 (denoted as CuTz‐1‐O_2_@F127) metal–organic framework (MOF) therapeutic platform is presented for enhanced PDT by simultaneously overcoming intracellular hypoxia and reducing GSH levels in the tumor. The Cu(I)‐based MOF is capable of a Fenton‐like reaction to generate ^•^OH and O_2_ in the presence of H_2_O_2_ under NIR irradiation. Meanwhile, the CuTz‐1‐O_2_@F127 nanoparticles (NPs) can release adsorbed O_2_, which further alleviates intracellular hypoxia. In addition, the Cu^I^ in CuTz‐1@F127 can react with intracellular GSH to reduce the excess GSH. In this way, the efficiency of PDT is greatly enhanced. After tail intravenous injection, the NPs show high antitumor efficacy through a synergistic effect under 808 nm laser irradiation. More importantly, the NPs are biodegradable. In vivo biodistribution and excretion experiments demonstrate that a total of nearly 90% of the NPs can be excreted via feces and urine within 30 d, which indicates significant prospects in the clinical treatment of cancers.

## 1 Introduction

Nowadays, humans are suffering from serious cancer attacks, and the incidence is still increasing.^1^ At present, the main methods for treating tumors include surgery,^2^ chemotherapy, radiotherapy (RT), gene therapy (GT), photodynamic therapy (PDT), photothermal therapy (PTT), immunotherapy, or the multimodal synergistic cancer therapy.^3^ PDT is an emerging treatment approved by the US Food and Drug Administration (FDA) that kills cancer cells via generating cytotoxic reactive oxygen species (ROS) by photosensitizer (PS) under light activation. It has the advantages of minimally invasive and good efficacy.^4^ Based on the different photochemical mechanism, PDT can be classified into two categories: type I PDT and type II PDT.[qv: 4d,e] Both type I and type II PDT involve the motivation of PS from ground singlet state to excited singlet state, and then to an electronically excited triplet state.[qv: 4d,f] For the most reported type II PDT process, the excited triplet state can convert triplet oxygen (^3^O_2_) into cytotoxic singlet oxygen (^1^O_2_).[qv: 4d] However, due to the rapid propagation of tumor tissues, the demand for oxygen (O_2_) far exceed the supply of O_2_, thus leading to aberrant growth of vascular systems, which hinders the diffusion of O_2_ and causes vicious cycles of hypoxia. Therefore, hypoxia originally pervades in solid tumors.^5^ Unfortunately, type II PDT system is highly dependent on O_2_ concentration and involves a sharp consumption of O_2_, which aggravates intracellular hypoxia and in reverse restrains the treatment effects of PDT.^6^

RETRACTED

To solve this problem, O_2_ self‐supply methods are widely used to elevate the concentration of O_2_ in tumors. A straightforward method is to transport O_2_ into tumor cells by utilizing O_2_ storage materials such as perfluorocarbon^7^ and metal–organic frameworks (MOFs).^8^ Another general strategy is to generate O_2_ in situ by catalysis to relieve hypoxia. The reported catalysts include catalase,^9^ MnO_2_,^10^ platinum(IV) diazido complexes,^11^ Pt nanozyme,^12^ MnFe_2_O_4_,^6^ carbon nitride,^13^ and so on. However, due to the severe hypoxia existing in malignant tumors, supplement of O_2_ is still less effective for type II PDT.^14^ Different from type II route, the type I reaction consists of the directly activated reactions between PS and substrates via a hydrogen‐ or electron‐transfer process and usually produces hydroxyl radicals (^•^OH) or superoxide radical (O_2_^•−^).[qv: 4c‐e,15] So far, a few nanostructures including ENBS‐B, LiYF_4_@SiO_2_@ZnO, TiO_2_‐ruthenium, Ce‐UCNPs, gold‐copper sulfide yolk–shell NPs, cyclometalated Ru(II) complexes, and Ti‐TBP nanoMOF have shown that type I PDT is highly effective under hypoxia.^14^, ^16^

Besides, hypoxia is particularly harmful; it can not only significantly increase the resistance to type II PDT and other therapies,^17^ but also trigger oncogenic transformation,[qv: 5a,18] which brings great difficulties to cancer treatment. Recent research showed that tumor hypoxia could cause DNA hypermethylation via reducing 10–11 translocation activity, whereas hypermethylation frequently inhibited the expression of tumor suppressor genes, thus promoting tumor progression.[qv: 5b] Another report revealed that hypoxia would promote the stable expression of hypoxia‐inducible factors (HIFs), and the resulting stabilization of HIF proteins in hypoxic cancer cells was thought to accelerate tumorigenesis.^18^ Therefore, overcoming hypoxia is highly desired for cancer therapy.

RETRACTED

Another key issue is that the overexpression of glutathione (GSH) in tumors is widespread, and the excess GSH would significantly reduce the cytotoxicity of ROS during the treatment of cancers, thus diminishing the efficacy of PDT.^19^ To date, the general strategies for solving this problem include the use of nanomaterials for intracellular oxidation reactions to reduce intracellular GSH levels.^19^

As a kind of burgeoning porous material, MOFs have been widely used for various applications.^20^ In particular, the hybrid materials with characteristic components can be easily functionalized and are excellent candidates for cancer treatment.^21^ Recently, Tang and co‐workers reported for the first time the use of Cu(II)‐based porphyrinic MOF with Cu^II^ as the active center to adsorb intracellular GSH for enhanced PDT.[qv: 21g] However, the researchers did not consider the severe hindrance of hypoxia to PDT. Moreover, the binding ability of Cu^II^ sites and sulfhydryl groups is not as strong as that of Cu^I^.[qv: 22a] Inspired by this observation, we design a biocompatible and biodegradable O_2_‐loaded CuTz‐1@F127 (denoted as CuTz‐1‐O_2_@F127) MOF therapeutic system for enhanced PDT by synchronously alleviating intracellular hypoxia and reducing GSH levels in tumors. It is worth noting that there was no previous report on overcoming hypoxia and reducing intracellular GSH at the same time. First, the CuTz‐1 MOF can act as a light‐activated photosensitizer (PS) to generate hydroxyl radicals (^•^OH) and O_2_ in the presence of hydrogen peroxide (H_2_O_2_), i.e., type I PDT, as shown in **Scheme** 1. In addition, the CuTz‐1@F127 can carry O_2_ molecules into cancer cells and adsorb intracellular GSH, alleviating both hypoxia and GSH overexpression at the same time, which can greatly promote the efficacy of PDT. The external F127 can enhance the biocompatibility of CuTz‐1‐O_2_. After tail intravenous (i.v.) injection, the CuTz‐1‐O_2_@F127 can accumulate in the tumor due to the enhanced permeability and retention (EPR) effect,^23^ and the NPs show high antitumor efficacy through synergistic effect under NIR irradiation. Besides, the preparation of CuTz‐1‐O_2_@F127 is facile, avoiding some complicated procedures. We endow the versatile capabilities of a single MOF material. More importantly, the CuTz‐1‐O_2_@F127 NPs are highly biocompatible and biodegradable. Biodistribution and excretion experiments show that in the early stage, CuTz‐1‐O_2_@F127 NPs mainly accumulate in the liver and spleen, and then are excreted via feces and urine along with the degradation of CuTz‐1‐O_2_@F127 NPs. After a month, a total of nearly 90% of the NPs can be excreted via feces and urine, which is of great importance for potential clinical application of nanomedicine.

RETRACTED

**Scheme 1:** a) Schematic illustration of preparation of CuTz‐1‐O_2_@F127 and b) for enhanced PDT.

## 2 Results and Discussions

### 2.1 Synthesis and Characterization of CuTz‐1@F127

It has been reported that CuTz‐1 could exhibit semiconductor‐like behavior and is capable of Fenton‐like reaction to generate ^•^OH in the presence of H_2_O_2_ under irradiation of Xe lamp.^24^ Moreover, it is attractive that CuTz‐1 exhibits continuous absorption from visible to near‐infrared (NIR) region (Figure S1, Supporting Information), which can be attributed to the intervalence charge‐transfer bands (IVCT) and the d–d transition. It is well known that IVCT is characteristic of mixed‐valence complexes. The absorption in the NIR region by CuTz‐1 could be related to the IVCT band involving Cu^I^ to Cu^II^ within the polymeric structure.^24^ So CuTz‐1 can be excited by 808 nm laser. Besides, the level of H_2_O_2_ in cancer cells is overexpressed, and many reports have shown that excess H_2_O_2_ inside the tumor can be used to overcome hypoxia in tumors.^14^, ^15^, ^16^ Thus, the CuTz‐1 MOF has great potential for the application of type I PDT under NIR laser excitation. As a proof‐of‐concept study, we first reduced the size of bulk CuTz‐1 to about 100 nm (Figure S2, Supporting Information) following a previous literature^24^ with slight modification, making it more suitable for biological applications. Then, an amphiphilic polymer F127 was coated to enhance the biocompatibility of CuTz‐1 (Scheme 1a).^25^ **Figure** 1a demonstrates that the morphology of CuTz‐1 did not change much before and after coating F127. The powder X‐ray diffraction (PXRD) pattern result (Figure 1b) confirms the structure of the NPs. The Fourier transform infrared spectra (FTIR) (Figure S3, Supporting Information) and thermogravimetric analysis (TGA) (Figure S4, Supporting Information) results demonstrate the successful coating of F127. TGA curves reveal that there was about 10 wt% of F127 coating on CuTz‐1. Additionally, the zeta potential, hydrodynamic size, and polydispersity index of CuTz‐1 and CuTz‐1@F127 suspended in DMEM culture medium containing 10% fetal bovine serum (FBS) are measured, respectively. As shown in Figure 1c,d and Figure S5 (Supporting Information), after coating F127, the mean zeta potential value changed from −5.6 ± 0.3 to −1.2 ± 0.1 mV, the dynamic light scattering (DLS) data showed the mean hydrodynamic size increased from 170.1 ± 11.5 to 186.4 ± 16.7 nm, and the polydispersity index decreased from 0.27 ± 0.03 to 0.14 ± 0.03, indicating the enhanced solubility and dispersity of CuTz‐1@F127 NPs in physiological environment. Besides, it should be noted that the particle sizes from DLS measurement are larger than the sizes observed from the corresponding SEM and TEM images (Figure S6, Supporting Information). The reason is that the DLS results give an average hydrodynamic particle size, while the SEM and TEM images show the dehydration morphology the NPs.[qv: 16d,26] Therefore, the size of the NPs obtained from the DLS result is larger than that observed from the SEM and TEM images.

RETRACTED

**Figure 1:** a) SEM and TEM images of CuTz‐1@F127. b) PXRD patterns of CuTz‐1 and CuTz‐1@F127. c) Zeta‐potentials of CuTz‐1 and CuTz‐1@F127. d) The average hydrodynamic size and the corresponding polydispersity index of CuTz‐1 and CuTz‐1@F127 suspended in DMEM culture medium containing 10% of fetal bovine serum.

### 2.2 Detection of Hydroxyl Radicals

The generation of ^•^OH was first examined by monitoring fluorescence enhancement of 3′‐(p‐aminophenyl) fluorescein (APF), which could selectively react with ^•^OH and become highly fluorescent.[qv: 16d] As shown in Figure S7 (Supporting Information), the obvious enhancement of APF fluorescence was observed in CuTz‐1@F127 phosphate buffer saline (PBS) solution in the presence of H_2_O_2_ upon 808 nm laser irradiation. Next, photodegradation experiment of rhodamine B (RhB) by CuTz‐1@F127 was carried out.^24^ As expected, the CuTz‐1@F127 could degrade RhB effectively in the presence of H_2_O_2_ upon laser irradiation (**Figure** 2a). Moreover, 2,7‐dichlorodihydrofluorescein diacetate (DCFH‐DA) was employed to monitor the intracellular ROS. DCFH‐DA can be hydrolyzed by esterase in cells and turn into DCFH, then the nonfluorescent DCFH can be oxidized to green‐fluorescent dichlorofluorescein (DCF) by ^•^OH.[qv: 16d] Figure S8 (Supporitng Information) shows that the cellular generation of ROS with CuTz‐1@F127 irradiated with an 808 nm laser (0.6 W cm^−2^) for 10 min. The green fluorescence indicated that ^•^OH was generated under the laser irradiation.

**Figure 2:** a) Degradation of RhB by CuTz‐1@F127 compared to TiO_2_ with or without GSH. b) The concentration of GSH in the supernatant solution after mixing with CuTz‐1@F127. c) The decrease of intracellular GSH with the increased concentrations of CuTz‐1@F127. d) HAADF image and EDS mapping result of a single CuTz‐1@F127@GSH nanoparticle. Scale bar is 100 nm. e) Oxygen adsorption–desorption isotherm of CuTz‐1@F127 at standard atmosphere pressure (760 mmHg) and room temperature (25 °C). f) Oxygen production and release performance of CuTz‐1‐O_2_@F127.

RETRACTED

### 2.3 In Vitro Study of Glutathione Reduction

Considering that excess GSH in cancer cells would weaken the effectiveness of PDT.^19^ We continue to investigate whether CuTz‐1@F127 can reduce intracellular GSH. First, after stirring with GSH, the CuTz‐1@F127 remained intact (Figure S9, Supporting Information). Then, we tested the GSH remaining in the supernatant using a reduced GSH assay kit. As shown in Figure 2b, although the size of GSH molecule is indeed larger than the aperture of CuTz‐1, due to the strong interaction between the coordination bonding of Cu^I^ sites and the sulfhydryl group,^22^ CuTz‐1@F127 could effectively reduce the content of GSH in the solution, far exceeding the ability of MOF‐2 to adsorb GSH.[qv: 21g] Nitrogen adsorption–desorption isotherm (Figure S10, Supporting Information) shows that BET surface area of CuTz‐1@F127 is 184.5 m^2^ g^−1^. However, after being mixed with GSH in aqueous solution, the value drops to 132.7 m^2^ g^−1^. The slight decrease demonstrates that GSH molecules combined with Cu^I^ site and occupied partial micropores of CuTz‐1@F127. The elemental mapping results (Figure 2d and Figure S11, Supporting Information) confirm that sulfur element uniformly distributed in the matrix, further demonstrating the CuTz‐1@F127 could adsorb GSH. In addition, in order to verify the effect of GSH on the oxidation ability of ^•^OH, GSH was added during the degradation experiment of RhB, and TiO_2_ was introduced for comparison, which is a well‐known photocatalyst.^27^ As illustrated in Figure 2a, both CuTz‐1@F127 and TiO_2_ showed excellent degradation efficiency for RhB under 808 nm and Xe lamp laser irradiation, respectively. However, when GSH was added, the degradation ability of TiO_2_ was seriously weakened, and CuTz‐1@F127 could still degrade nearly 70% of RhB. This result demonstrates that CuTz‐1@F127 could reduce GSH effectively and keep the lethality of ^•^OH.

### 2.4 In Vitro Study of Oxygen Generating

Notably, MOFs are good candidates for O_2_ storage.^28^ In particular, the Cu‐based MOFs possess ultrahigh O_2_ storage capacities due to coordinatively unsaturated Cu sites. In view of this, we tested the O_2_ adsorption capacity of CuTz‐1@F127. Oxygen adsorption–desorption isotherm (Figure 2e) reveals that CuTz‐1@F127 could adsorb up to 400 µmol g^−1^ of O_2_ at standard atmospheric pressure and room temperature. After being immersed in an O_2_ atmosphere, CuTz‐1‐O_2_@F127 was obtained (Scheme 1a). To demonstrate the O_2_ production and release performance of CuTz‐1‐O_2_@F127, we measured O_2_ concentration under 808 nm laser irradiation. As shown in Figure 2f, an increase of O_2_ concentration was observed in CuTz‐1@F127 PBS solution at a low H_2_O_2_ concentration, demonstrating the production of O_2_ during the Fenton‐like reaction. Because there are electrons and holes occurring during the conversion of Cu^I^ to Cu^II^ stimulated by NIR, which may lead to release of the adsorbed O_2_.^24^ Therefore, the CuTz‐1‐O_2_@F127 NPs can release adsorbed O_2_ within cancer cells, further alleviating intracellular hypoxia. Ultimately, both the generated and released O_2_ can overcome intracellular hypoxia, which plays an auxiliary role in the PDT.

RETRACTED

### 2.5 Cell Studies: Cellular Uptake, Biocompatibility, and Photocytotoxicity

In vitro experiments were further conducted to investigate the antitumor efficacy of CuTz‐1‐O_2_@F127. First, inverted fluorescence microscopy images revealed that the NPs could be endocytosed by 4T1 cells (mouse breast cancer cells) within 4 h (Figure S12, Supporting Information). Then, L929 cells (mouse fibroblast cells), HeLa cells and 4T1 cells were chosen to test the biosafety via the MTT (3‐(4,5‐dimethylthiazol‐2‐yl)‐2,5‐diphenyltetrazolium bromide) cell‐viability assay. As shown in **Figure** 3a, although the concentration of CuTz‐1‐O_2_@F127 was as high as 200 × 10^−6^ m, the viability of L929 cells was still nearly 100% after incubated for 24 h, indicating the CuTz‐1‐O_2_@F127 is highly biocompatible to normal cells. Intriguingly, the activity of HeLa and 4T1 cancer cells decreased when the concentration of CuTz‐1‐O_2_@F127 exceeded 100 × 10^−6^ m. This is because CuTz‐1‐O_2_@F127 can adsorb intracellular GSH, and the decrease of GSH affects the normal growth of cancer cells, leading to the difference in the viability of cancer cells and normal cells.[qv: 21g] Next, the PDT effectiveness of CuTz‐1@F127 and CuTz‐1‐O_2_@F127 incubating with 4T1 cells in both hypoxic and normoxic conditions was measured. The viability of 4T1 cells was examined by MTT assay after CuTz‐1@F127 + light and CuTz‐1‐O_2_@F127 + light treatment and further incubated for 24 h. As displayed in Figure 3b, hypoxia‐treated groups exhibited higher cell survival than those of normoxia under irradiation. This result suggests that intracellular hypoxia facilitates proliferation of cancer cells,^12^, ^18^ reinforcing the importance of overcoming hypoxia during tumor treatment. As expected, the therapeutic effect of CuTz‐1‐O_2_@F127 + light treated group under hypoxia was similar to that under normoxic condition, and the treatment effect increased along with the concentration of CuTz‐1‐O_2_@F127. The flow cytometric analyses (Figure S13, Supporting Information) further proved that the CuTz‐1‐O_2_@F127 + light group showed the lowest percentage of cell survival (about 21.1%).

RETRACTED

**Figure 3:** a) In vitro cell viability data of CuTz‐1‐O_2_@F127 against L929, HeLa, and 4T1 cells after incubation for 24 h. b) In vitro PDT effect of 4T1 cells against CuTz‐1@F127 and CuTz‐1‐O_2_@F127 under 808 nm laser irradiation in hypoxic or normoxic conditions after 24 h incubation. c) ROS and hypoxia generation in cells after incubation with CuTz‐1@F127 or CuTz‐1‐O_2_@F127 with or without 808 nm laser irradiation. Fluorescence images of the cells stained with ROS and hypoxia probe. Cell nuclei were stained by DAPI. Scale bar is 50 µm. d) Live‐dead staining images of 4T1 cells treated with PBS (control), PBS + light, CuTz‐1@F127, CuTz‐1‐O_2_@F127, CuTz‐1@F127 + light, and CuTz‐1‐O_2_@F127 + light, respectively, under hypoxia. Scale bar is 200 µm.

### 2.6 Intracellular Detection of ROS and Hypoxia

We further used the ROS‐ID hypoxia/oxidative stress detection kit to explore intracellular ROS and hypoxia. As shown in Figure 3c, as control groups, there was no ROS production without light irradiation. However, strong ROS signals were detected with 808 nm laser irradiation under both hypoxia and normoxia, indicating the type I PDT process is capable of producing large amounts of ^•^OH even under hypoxia. Moreover, after NIR irradiation, the CuTz‐1@F127 + light and CuTz‐1‐O_2_@F127 + light group treated cells under hypoxia showed weaker red fluorescence than that of without irradiation, demonstrating that CuTz‐1@F127 can produce O_2_ in the cells under NIR irradiation, and the CuTz‐1‐O_2_@F127 + light group showed a more weaker red fluorescence than the CuTz‐1@F127 + light group, suggesting CuTz‐1‐O_2_@F127 can further release the O_2_ it carries to relieve hypoxia in cancer cells.

### 2.7 Live/Dead Cell Staining Analysis

To further examine the phototoxicity of the CuTz‐1 MOF system under hypoxia, the live (green fluorescence) and dead cells (red fluorescence) were distinguished by a Calcein‐AM/PI double stain kit. As shown in Figure 3d, as a comparison, all cells untreated or cultivated with PBS + light, CuTz‐1@F127 and CuTz‐1‐O_2_@F127, the cells showed green fluorescence, implying ignorable cell damage. Upon 808 nm laser irradiation, only small green fluorescence was observed in CuTz‐1@F127 treated group, suggesting most cells were dead. All cells treated with CuTz‐1‐O_2_@F127 + light were dead and stained with red fluorescence. These results further suggest the superior therapeutic efficacy of CuTz‐1‐O_2_@F127 to overcome hypoxia for enhanced PDT of cancer cells.

RETRACTED

### 2.8 In Vivo Tumor Inhibition Ability

Encouraged by the effective PDT effect in vitro, we further investigated the therapeutic effect of CuTz‐1‐O_2_@F127 in vivo on the 4T1 tumor‐bearing mice. Six groups of female Balb/c mice bearing 4T1 tumors (*n* = 5) were respectively treated by tail i.v. injection at a dose of 20 mg kg^−1^ with PBS as control, PBS + light, CuTz‐1@F127, CuTz‐1‐O_2_@F127, CuTz‐1@F127 + light or CuTz‐1‐O_2_@F127 + light. The body weights and tumor sizes were measured every 2 d. **Figure** 4a shows the body weights of mice in all groups increased gradually along with time, suggesting that these operations have little side effects on mice. Figure 4b shows the therapeutic effect on tumors over time. Compared with control groups, both CuTz‐1@F127 and CuTz‐1‐O_2_@F127 treated groups showed a certain effect on inhibiting tumors. This is because the CuTz‐1@F127 can reduce the level of GSH in tumors (Figure 4c), thereby affecting the normal growth of cancer cells.^45^ Finally, the tumors treated with CuTz‐1@F127 + light and CuTz‐1‐O_2_@F127 + light were efficiently inhibited. Moreover, due to more O_2_ supplements, the CuTz‐1‐O_2_@F127 + light group showed the best tumor suppression. The above results demonstrate that the O_2_‐loaded MOF therapeutic system can realize effective tumor destruction under 808 nm laser irradiation. After 14 d of treatment, all mice were sacrificed and tumors were excised and weighed. Figure 4d and Figure S14 (Supporting Information) show that the tumor growth in CuTz‐1‐O_2_@F127 + light group was distinctly inhibited after the enhanced PDT. In situ hematoxylin and eosin (H&E) staining of tumor tissues was executed to test the efficacy. As shown in Figure 4e, the obvious necrosis of tumor tissues can be observed in both CuTz‐1@F127 + light and CuTz‐1‐O_2_@F127 + light groups, indicating the lethality of ^•^OH. Meanwhile, the H&E staining images of the main organs including liver, spleen, lung, kidney and heart treated with CuTz‐1‐O_2_@F127, CuTz‐1@F127 + light, CuTz‐1‐O_2_@F127 + light as well as control group were also tested (Figure S15, Supporting Information). As expected, no obvious tissue damages can be found, indicating the good biosafety of CuTz‐1‐O_2_@F127.

**Figure 4:** a) The body weights and b) the relative tumor volumes of mice after treated with PBS (control), PBS + light, CuTz‐1@F127, CuTz‐1‐O_2_@F127, CuTz‐1@F127 + light, and CuTz‐1‐O_2_@F127 + light, respectively. c) Measurement of GSH content within the tumors by using a reduced GSH assay kit as a function of time. The i.v. injection dose is 20 mg kg^−1^. d) In vivo antitumor efficacy of CuTz‐1‐based nanoplatform on 4T1 tumor‐bearing Balb/c mice. e) Hematoxylin and eosin (H&E) staining of tumor slices for all groups. Error bars indicated the standard deviations, *N* = 5.

RETRACTED

### 2.9 In Vivo Long‐Term Toxicity, Biodistribution, and Excretion Studies

In addition, the long‐term toxicity and in vivo biodistribution of CuTz‐1‐O_2_@F127 were carried out on Balb/c mice via i.v. injection of NPs. As shown in Table S1 (Supporting Information), serum biochemistry data show that there were no major parameter differences between the treatment group and the control group, including the creatine kinase (CK) for heart function; blood urea (BUN) and serum creatinine (CRE) for renal function; alanine aminotransferase (ALT), aspartate aminotransferase (AST) and alkaline phosphatase (ALP) for hepatic function. Moreover, in order to determine the in vivo biodistribution of CuTz‐1‐O_2_@F127 NPs, the main organs and tumors of all mice were collected at regular intervals after tail i.v. injection. The copper concentrations were determined by inductively coupled plasma‐mass spectrometer (ICP‐MS). As shown in **Figure** 5a, within the first 12 h after i.v. injection, the NPs were mainly absorbed by liver and spleen. Due to the EPR effect,^23^ a large amount of NPs could accumulate at the tumor site and reach the maximum at about 24 h. Then the NPs decreased in the tested organs with the prolonged time. We further investigated the excretion of NPs in mice. Interestingly, as shown in Figures S16 and S17 (Supporting Information), SEM and PXRD data reveal that the CuTz‐1‐O_2_@F127 started decomposing when immersed in PBS solution on the fifth day. On the 10 day, CuTz‐1‐O_2_@F127 completely lost its morphology and crystal structure. This result offers great possibility for CuTz‐1‐O_2_@F127 to be completely eliminated from the body. So we further measured the amount of Cu in feces and urine collected from CuTz‐1‐O_2_@F127‐injected mice at different intervals. In the early time, NPs accumulated in liver would be mainly excreted by bile into feces. After a week, the degraded NPs could be excreted through kidney to form urine (Figure 5b).^29^ At 14th day, the NPs reached a maximum with the excretion of urine. Thereafter, the discharge amount is gradually reduced, and after 30 d, the NPs were discharged at a high rate of ≈90% through feces and urine. This phenomenon indicates that although CuTz‐1 is stable in GSH aqueous solution, it is biodegradable due to the complex TME and can be excreted out of the body, which greatly demonstrates the biodegradablity of CuTz‐1‐O_2_@F127.

**Figure 5:** a) The in vivo biodistribution of Cu after i.v. injection with CuTz‐1‐O_2_@F127 at different time. b) Excretion percentages of CuTz‐1‐O_2_@F127 in feces and urine of mice at different time after tail i.v. injection.

RETRACTED

## 3 Conclusion

In summary, we for the first time develop a CuTz‐1‐O_2_@F127 therapeutic platform for enhanced PDT of cancers. The fabrication of such nanoscale MOF therapeutic agent is simple and straightforward. This research demonstrates the use of CuTz‐1‐O_2_@F127 as a potential PDT agent, which possesses excellent ability to produce ^•^OH and overcome intracellular hypoxia, as well as the ability to reduce intracellular GSH levels. Although the expatiation of type I PDT mechanisms, especially whether O_2_ plays a role, are still debatable.[qv: 4e] Our both in vitro and in vivo experiments show that overcoming hypoxia can enhance the PDT. More importantly, the CuTz‐1‐O_2_@F127 can be excreted out of mice body at a high rate of ≈90% through feces and urine after a month, which is of great importance for potential clinical application of nanomedicine.

## 4 Experimental Section

*Chemicals and Materials*: 3,5‐Diphenyl‐1,2,4‐triazole (3,5‐Ph_2_‐tzH) was purchased from Jilin Province In‐depth Research Technology Co., Ltd. Tetrakis (acetonitrile) copper(I) tetrafluoroborate (Cu(CH_3_CN)_4_BF_4_) were purchased from Tokyo Chemical Industry Co., Ltd. (TCI). Methanol, concentrated hydrochloric acid (HCl, 36%), concentrated nitric acid (HNO_3_, 65%–68%), hydrogen peroxide (H_2_O_2_, 30%), and 3′‐(p‐aminophenyl) fluorescein (APF) were purchased from Beijing Chemical Factory. Pluronic F127 was purchased from Sigma‐Aldrich. 3‐(4,5‐dimethylthiazol‐2‐yl)‐2,5‐diphenyltetrazolium bromide (MTT), 4,6‐diamino‐2‐phenylindole (DAPI), titanium dioxide (TiO_2_), glutathione (GSH), and fluorescein isothiocyanate (FITC) were purchased from Shanghai Aladdin Bio‐Chem Technology Co., Ltd. HS‐OEG‐NH_2_ was purchased from Shenzhen Xing Jia Feng Science and Technology Development Co., Ltd. Calcein‐AM/PI Double Stain Kit was purchased from Beyotime Biotechnology. Annexin V‐FITC/PI double‐staining apoptosis detection kit was purchased from Shanghai BestBio. Reduced glutathione (GSH) assay kit was purchased from Beijing Solarbio Science & Technology Co., Ltd. ROS‐ID hypoxia/oxidative stress detection kit was purchased from Enzo Life Sciences. All reagents were used as purchased from commercial sources without further purification. Deionized water (18.2 MΩ) was used in all experiments and to prepare all buffers.

*General Analytical Techniques*: Power X‐ray diffraction (XRD) measurements were performed on a D8 focus diffractometer with graphite monochromatized Cu Kα radiation (λ = 0.15405 nm). Thermogravimetric analysis (TGA) was recorded on Thermal Analysis Instrument (SDT 2960, TA Instruments, New Castle, DE) with a heating rate of 10° min^−1^ in a nitrogen flow of 100 mL min^−1^ from room temperature to 800 °C. The morphology of the samples was characterized by a field‐emission scanning electron microscope (FE‐SEM, S‐4800, Hitachi) equipped with an energy‐dispersive X‐ray (EDX) spectrometer. Transmission electron microscopy (TEM) images were obtained on a FEI Tecnai G2 S‐Twin with a field emission gun operating at 200 kV. Fourier transform infrared spectra (FT‐IR) were measured on a Vertex PerkinElmer 580BIR spectrophotometer (Bruker) with KBr pellet technique. The UV–vis adsorption spectra were measured on a Hitachi U‐3100 spectrophotometer. Nitrogen absorption/desorption analysis was measured on an Autosorb IQ instrument. The samples were fully exchanged with ethanol, and degassed at 150 °C for 8 h before gas adsorption measurement. Concentrations of Cu were measured by the inductively coupled plasma‐mass spectrometer (ICP‐MS). Dynamic light scattering (DLS) experiment was measured by Malvern Zeta Sizer‐Nano ZS90 instrument at 25 °C.

RETRACTED

*Synthesis of CuTz‐1@F127 and CuTz‐1‐O_2_@F127 Nanoparticles (NPs)*: A precursor solution was first prepared by mixing 3,5‐Ph2‐tzH (5.5 mg, 0.025 mmol) in 1.0 mL of methanol and 0.1 mL of deionized water. Then, Cu(CH_3_CN)_4_BF_4_ (15 mg, 0.05 mmol) dissolved in 1.0 mL of methanol was added into the above solution. The mixture was then stirred at room temperature for 3 h. Afterward, the white powder was collected by centrifugation, washed three times with methanol. To connect fluorescent FITC to the surface of the CuTz‐1 NPs, CuTz‐1 (5.0 mg) was first mixed with HS‐OEG‐NH_2_ (10 mg) in 2.0 mL of deionized water for 10 h at room temperature, then 1.0 mg of FITC was added and the mixtures were further stirred overnight. Finally, the yellow products were collected by centrifugation and washed three times with deionized water. To coat pluronic F127 on the surface of CuTz‐1, pluronic F127 was first dissolved in methanol (10 mg mL^−1^) and added into CuTz‐1 methanol solution (concentration of CuTz‐1 is at 1 mg mL^−1^). After ultrasonic dispersion, the solvent was removed by rotary evaporator at 40 °C for 5 h, the dried CuTz‐1@F127 was obtained. After being immersed in an oxygen atmosphere for 6 h, the CuTz‐1‐O_2_@F127 was obtained.

*Degradation Experiment of CuTz‐1@F127 NPs*: The CuTz‐1@F127 NPs were immersed in PBS solution (pH 6.5 and pH 7.4) and taken out at intervals for SEM and PXRD test.

*Hydroxyl Radical Detection*: Hydroxyl radicals were specifically determined by 3′‐(p‐aminophenyl) fluorescein (APF) assay. 100 × 10^−6^ m of CuTz‐1@F127 phosphate buffer saline (PBS) solution in the presence of 1.0 × 10^−3^ m of H_2_O_2_ was gently mixed with 80 µL of APF solution(10 × 10^−3^ m). The resulting mixture was exposed to an 808 nm laser (0.6 W cm^−2^) irradiation for 10 min, followed by 2 h of incubation at room temperature. APF fluorescence emission spectra in the range of 480–600 nm were collected with an excitation wavelength of 455 nm.

RETRACTED

*Photodegradation Experiment of RhB*: The photocatalytic activity of CuTz‐1@F127 was evaluated by photodegradation of RhB in aqueous solution under 808 nm laser irradiation (0.6 W cm^−2^) at room temperature. For TiO_2_ photocatalysis, a Xenon lamp with a fiber optic (1.0 W cm^−2^) was used. Specifically, the photocatalyst CuTz‐1@F127 (1.0 mg) was dispersed in 2.0 mL of aqueous solution containing 1.0 ppm of RhB and 1.0 × 10^−3^ m of H_2_O_2_. The concentration of TiO_2_ was 5.0 mg mL^−1^. The concentration of RhB was determined by UV–vis spectroscopy. To study the effects of GSH, 1.0 × 10^−3^ m of GSH was added additionally and the mixture was stirred for 24 h before irradiation.

*Intracellular ROS Detection*: For intracellular ROS detection, 4T1 cells were seeded in 12‐well plates and incubated for 24 h. Then, CuTz‐1@F127 was added into each well with the particle concentration of 50 × 10^−6^ m after 4 h, the cells were exposed to 808 nm light (0.6 W cm^−2^) for 5 min. After incubated for another 1 h, DCFH‐DA in DMEM was added into wells and kept for 30 min. Then, cells were washed with PBS for several times to abandon noninternalized NPs. The fluorescence images of different cell groups were acquired using inverted fluorescence microscope.

*Detection of the Reduced GSH Both In Vitro and In Vivo*: The content of reduced GSH was determined directly by a Reduced Glutathione Assay Kit. For in vitro testing, GSH (1.0 × 10^−3^ m) was mixed with CuTz‐1@F127 (200 × 10^−6^ m) for 12 h under vibration. Then, the solution was centrifuged and the supernatant was tested according to the manufacturer's protocol. For in vivo testing, 24 tumor‐bearing Balb/c mice were divided into two groups equally. One group of mice were intravenously injected CuTz‐1‐O_2_@F127 at a dose of 20 mg kg^−1^. The other group was as a control. The tumors of all mice were collected at regular intervals and the content of reduced GSH was tested according to the manufacturer's protocol.

*The Measurement of the Generated and Released Oxygen*: To demonstrate the oxygen production and release performance of CuTz‐1‐O_2_@F127, the NPs (10 mg mL^−1^) were immersed in 5.0 mL of deoxygenated PBS solution (pH 6.5) in the presence of H_2_O_2_ (0.5 × 10^−3^ m) under 808 nm laser irradiation. Then, the amount of dissolved oxygen was determined by a portable dissolved oxygen meter every minute.

RETRACTED

*Cell Culture*: Mouse fibroblast cells (L929 cells), mouse breast cancer cell (4T1 cells), and HeLa cells were cultured in high glucose DMEM supplemented with 10% fetal bovine serum (FBS), 1% (v/v) penicillin/streptomycin at 37 °C under 5% CO_2_/95% air. For hypoxic experiments, 4T1 cells were cultured under 5% CO_2_/94% N_2_/1% O_2_.

*Cellular Uptake*: 4T1 cells (10^5^ cells per well) were seeded in six‐well culture plate and grown overnight. 2.0 mL of DMEM medium containing CuTz‐1‐FITC@F127 (50 × 10^−6^ m) was added to each well of the six‐well plate. After the incubation for 10 min and 4 h at 37 °C, respectively, 4T1 cells were washed by PBS, fixed with polyformaldehyde aqueous solution (4%; 1 mL per well), then washed with PBS again. Finally, 1.0 mL of DAPI solution (10 µg mL^−1^ in PBS) was added for staining. Afterwards, the cells were washed by PBS for another two times and detected by an inverted fluorescence microscope.

*Cytotoxicity Assays*: L929 cells, HeLa cells, and 4T1 cells were seeded in 96‐well plates and incubated for 24 h. Afterwards, CuTz‐1‐O2@F127 at a concentration of 25 × 10^−6^, 50 × 10^−6^, 100 × 10^−6^, 150 × 10^−6^ and 200 × 10^−6^ m was added, respectively, and incubated with cells for 24 h. Finally, MTT solution (20 µL, 5 mg mL^−1^) was added into each well. The 96‐well plates were incubated for another 4 h before replacing the original culture medium with 150 µL of DMSO. The surviving rate of 4T1 cells was figured out using a microplate reader.

*In Vitro PDT of CuTz‐1@F127 and CuTz‐1‐O_2_@F127*: 4T1 cells harvested in a logarithmic growth phase were seeded in 96‐well plates at a density of 5 × 10^4^ cells per well and incubated in DMEM for 24 h at 37 °C under 5% CO_2_/95% air for normoxic experiment and 5% CO_2_/94% N_2_/1% O_2_ for hypoxic experiment, respectively. The cells were incubated with different concentrations of CuTz‐1@F127 and CuTz‐1‐O_2_@F127 (0 × 10^−6^, 6.25 × 10^−6^, 12.5 × 10^−6^, 25 × 10^−6^, 50 × 10^−6^, 100 × 10^−6^ m) for another 4 h. Then, the plates were irradiated with 808 nm laser at a power density of 0.6 W cm^−2^ for 20 min. (After 10 min of irradiation, it was interrupted for 5 min and then irradiated for another 10 min.) After that, cells were placed in a cell culture box and further incubated for 24 h. The evaluation of the photodynamic cytotoxicity was performed by MTT assay as described above.

*Annexin Flow Cytometry*: For flow cytometry, 4T1 cells were seeded into six‐well culture plates and treated with (a) PBS + light; (b) CuTz‐1‐O_2_@F127, (100 × 10^−6^ m of Cu); (c) CuTz‐1@F127 + light (100 × 10^−6^ m of Cu); (d) CuTz‐1‐O_2_@F127 + light (100 × 10^−6^ m of Cu). After 808 nm light irradiation (0.6 W cm^−2^; 20 min), all 4T1 cells were incubated for further 12 h at 37 °C in the dark. To obtain a single cell suspension, the 4T1 cells were washed by trypsinization and PBS continuously. Then, the cells were stained by the annexin V‐FITC and PI staining kit. A FACS Calibur flow cytometer (BD Biosciences) was used to detect the induction of apoptosis in 4T1 cells.

RETRACTED

*Intracellular ROS and Hypoxia Analysis*: 4T1 cells were cultured in a six‐well culture plate (5 × 10^4^ cells per well) and grown in hypoxic or normoxic environment for 24 h. Then, cells were treated with CuTz‐1 @F127, CuTz‐1@F127 + light or CuTz‐1‐O_2_@F127 + light and then administrated with the ROS‐ID Hypoxia/Oxidative stress detection kit according to the manufacturer's instructions. After 20 min, the cells were washed twice and exposed to 808 nm laser irradiation for 5 min. After that, cells were washed with PBS, stained by DAPI, and observed by inverted fluorescence microscopy.

*Live/Dead Cell Staining Analysis*: 4T1 cells were cultured in a six‐well culture plate (1 × 10^5^ cells per well) and grown in hypoxic environment for 24 h. Then the cells were treated with PBS (control), PBS + light, CuTz‐1@F127, CuTz‐1‐O_2_@F127, CuTz‐1@F127 + light and CuTz‐1‐O_2_@F127 + light, respectively, followed by another 15 h of incubation. After the treatment, the cells were stained by 400 µL of the mixture of Calcein‐AM (1 × 10^−6^ m) and propidium iodide (PI) (1 × 10^−6^ m) for 20 min. After being washed three times, the cells were visualized using an inverted fluorescence microscopy.

*In Vivo Antitumor Efficacy Experiment*: Female Balb/c mice (about 24 g) were purchased from the Center of Experimental Animals, Jilin National Regulation of China for Care and Use of Laboratory Animals. All the animal experiments were carried out in accordance with the relevant laws. The tumor models were generated by subcutaneous injection of 1 × 10^6^ 4T1 cells in 0.1 mL PBS into the left axilla of the mice. The mice were used when the tumor volume reached about 100 mm^3^. For in vivo anticancer experiment, 30 tumor‐bearing mice were divided into six groups (control, PBS + light, CuTz‐1@F127, CuTz‐1‐O_2_@F127, CuTz‐1@F127 + light and CuTz‐1‐O_2_@F127 + light treated groups). NPs were injected through tail vein two times on day 1 and 7, respectively. For the irradiation groups, the mice were irradiated with 808 nm laser at a power density of 0.6 W cm^−2^ for 20 min after 24 h of the injection. (After 10 min of irradiation, it was interrupted for 5 min and then irradiated for another 10 min.) The body weight and tumor volumes of each mouse were recorded every 2 d. The main organs and tumor tissues of the mice were isolated and fixed for further histological examination. The tumor volume (*V*) was determined by measuring length (*L*) and width (*W*), and calculated as *V* = (*W* ^2^ × *L*)/2. The relative tumor volumes were calculated for each mouse as *V*/*V*_0_ (*V*_0_ is the tumor volume when the treatment is initiated). It is worth noting that no mice died during the experiments.

RETRACTED

*Toxicology Evaluation of CuTz‐1‐O_2_@F127 NPs*: Healthy Balb/c mice were intravenously injected with PBS (control group) and CuTz‐1‐O_2_@F127 NPs at a dose of 20 mg kg^−1^ (test group), respectively. After injection at different times (day 1, day 7, and day 14), mice were euthanized and then the blood was collected for biochemistry analysis.

*In Vivo Biodistribution and Excretion of CuTz‐1‐O_2_@F127 NPs*: To determine the biodistribution of CuTz‐1‐O_2_@F127 NPs, mice after i.v. injection with CuTz‐1‐O_2_@F127, major organs and tissues (heart, liver, spleen, lung kidney, and tumor) from Balb/c mice (*n* = 3) were collected at a certain time interval. Next, the collected organs were wet‐weighted and dissolved in chloroazotic acid under heating at 60 °C for 12 h. After each sample was diluted with deionized water to 10 mL, ICP‐MS was used to measure Cu concentrations in different samples. To study the excretion of CuTz‐1‐O_2_@F127 NPs, mice after i.v. injection with CuTz‐1‐O_2_@F127 were kept in metabolic cages to collect urine and feces. The obtained urine and feces were digested by chloroazotic acid and measured by ICP‐MS.

## Conflict of Interest

The authors declare no conflict of interest.

## Supporting information

Supplementary
